The article "Echocardiography, Spirometry, and Systemic Acute-Phase Inflammatory Proteins in Smokers with COPD or CHF: An Observational Study" was published in 2013. Journal: PLoS One.

# Echocardiography, Spirometry, and Systemic Acute-Phase Inflammatory Proteins in Smokers with COPD or CHF: An Observational Study

**DOI:** 10.1371/journal.pone.0080166

**Published:** 2013-11-11

**Authors:** Bianca Beghé, Alessia Verduri, Barbara Bottazzi, Mariarita Stendardo, Alessandro Fucili, Sara Balduzzi, Chiara Leuzzi, Alberto Papi, Alberto Mantovani, Leonardo M. Fabbri, Claudio Ceconi, Piera Boschetto

**Affiliations:** 1 Department of Medical and Surgical Sciences, University of Modena & Reggio Emilia, Modena, Italy; 2 Laboratory of Research in Immunology and Inflammation, Humanitas Clinical and Research Center, Rozzano, and Department of Translational Medicine, University of Milan, Milan, Italy; 3 Department of Medical Sciences, University of Ferrara, Ferrara, Italy; VU University Medical Center, Netherlands

## Abstract

Chronic obstructive pulmonary disease (COPD) and chronic heart failure (CHF) may coexist in elderly patients with a history of smoking. Low-grade systemic inflammation induced by smoking may represent the link between these 2 conditions. In this study, we investigated left ventricular dysfunction in patients primarily diagnosed with COPD, and nonreversible airflow limitation in patients primarily diagnosed with CHF. The levels of circulating high-sensitive C-reactive protein (Hs-CRP), pentraxin 3 (PTX3), interleukin-1β (IL-1 β), and soluble type II receptor of IL-1 (sIL-1RII) were also measured as markers of systemic inflammation in these 2 cohorts. Patients aged ≥50 years and with ≥10 pack years of cigarette smoking who presented with a diagnosis of stable COPD (n=70) or stable CHF (n=124) were recruited. All patients underwent echocardiography, N-terminal pro-hormone of brain natriuretic peptide measurements, and post-bronchodilator spirometry. Plasma levels of Hs-CRP, PTX3, IL-1 β, and sIL-1RII were determined by using a sandwich enzyme-linked immuno-sorbent assay in all patients and in 24 healthy smokers (control subjects). Although we were unable to find a single COPD patient with left ventricular dysfunction, we found nonreversible airflow limitation in 34% of patients with CHF. On the other hand, COPD patients had higher plasma levels of Hs-CRP, IL1 β, and sIL-1RII compared with CHF patients and control subjects (p < 0.05). None of the inflammatory biomarkers was different between CHF patients and control subjects. In conclusion, although the COPD patients had no evidence of CHF, up to one third of patients with CHF had airflow limitation, suggesting that routine spirometry is warranted in patients with CHF, whereas echocardiography is not required in well characterized patients with COPD. Only smokers with COPD seem to have evidence of systemic inflammation.

## Introduction

Chronic obstructive pulmonary disease (COPD) and chronic heart failure (CHF) are important causes of morbidity and mortality worldwide, particularly in the elderly [1,2]. Despite the fact that COPD and CHF present a major challenge for healthcare providers and share common risk factors—in particular, cigarette smoking—few studies have addressed the association of CHF and COPD and its impact on patient management and prognosis in well-characterized patient cohorts [3].

Cigarette smoking is the major risk factor for COPD and cardiovascular diseases. It causes systemic inflammation, oxidative stress, increased circulating concentration of inflammatory cytokines, and changes in endothelial functions. Low-grade systemic inflammation has been proposed to be the common substrate of chronic diseases such as COPD and CHF, and thus it is a possible link between these diseases and their comorbidities [4].

C-reactive protein (CRP) is the most established marker of systemic inflammation, plays an important role in COPD [5], and is involved, although to a lesser extent, also in CHF [6]. Recently, another acute phase inflammatory protein of the pentraxin family (PTX3) has been proved to be linked to the severity and prognosis of CHF [7]. PTX3 is a component of the humoral arm of the innate immune system which, unlike CRP, is produced also at the site of inflammation [7]. We speculated that examining and comparing plasma levels of CRP and PTX3 might add information on the role of systemic inflammation in COPD and CHF. As interleukin-1β (IL-1 β) is a pro-inflammatory cytokine and one of the main inducer of PTX3 [7], it was included in the cytokines to be measured. Since the decoy receptor sIL-1RII plays a key role in downing the action of IL-1 β [8], its plasma level has also been determined. 

Recognition of comorbid heart failure in COPD patients and of COPD symptoms in CHF patients is hampered by similarities in signs and symptoms, in particular, dyspnea. Moreover, even though it is well known that spirometry is essential to establish the diagnosis of COPD, and echocardiography is essential for the diagnosis of CHF, epidemiological data suggest an under-use in clinical practice of both measurements in smokers [9]. Indeed, in most retrospective studies reporting the coexistence of COPD and CHF, the diagnoses were not based on spirometry and echocardiography [10,11]. Thus, the aims of our study were 1) to assess the occurrence of CHF by echocardiography in well-characterized, spirometrically documented smokers with COPD; 2) to assess the occurrence of COPD by spirometry in well-characterized smokers with CHF; and 3) to assess the degree of systemic inflammation by measuring circulating high-sensitive C-reactive protein (Hs-CRP), PTX3, IL-1 β, and soluble type II receptor (decoy receptor) of IL-1 (sIL-1RII) in both cohorts.

## Materials and Methods

This was a two-center observational study.

### Study Subjects

A total of 218 subjects were studied: 70 COPD patients, 124 CHF patients, and 24 healthy smokers. Patients aged ≥50 years who had a smoking history of ≥10 pack years were enrolled at the Respiratory Unit of the University Hospital of Modena and at the Heart Failure Centre of the University Hospital of Ferrara, respectively, between July 2009 and September 2010. The control group of 24 age-matched healthy smokers (≥10 pack years) had no known cardiac or respiratory diseases or symptoms and were recruited from the same outpatient clinics.

COPD patients had been free from exacerbations for 4 weeks, and CHF patients had been on stable medication for 3 months.

The study conformed to the Declaration of Helsinki and was approved by the institutional ethics committees of each participating university hospital (Comitato Etico Provinciale di Ferrara and Comitato Etico Provinciale di Modena). All participants provided signed informed consent before recruitment (ClinicalTrials.gov number, NCT01114386).

Demographic/morphological data and results from body mass index (BMI), spirometry, Charlson comorbidity index, 6-min walk test (6MWT), basic biochemistry, N-terminal pro-hormone brain natriuretic peptide (NT-proBNP), HsCRP, PTX3, IL-1 β, and sIL-1RII were obtained from all study participants. COPD and CHF patients also underwent electrocardiography and echocardiography. Subsets of data collected from patients with CHF were reported previously [12].

### Sample Collection

Blood samples were obtained from all study subjects for assessment of plasma concentrations of PTX3, IL-1 β, and sIL-1RII. Blood samples were centrifuged at 1,500 x *g* for 10 min at 7 °C. Plasma aliquots were stored at -80 °C until assayed.

### Clinical and Functional Assessment

Spirometry (Biomedin, Padova, Italy) and the 6MWT were performed according to current international guidelines [13,14].

Echocardiography was carried out by following a standard protocol that included the measurements and the validated diagnostic criteria recommended by the European Society of Echocardiology [2].

### Measurements of PTX3, IL-1 β, and sIL-1RII

Plasma levels of PTX3 and sIL-1RII were measured by in-house sandwich ELISA as previously described [15,16]. Detection limit was 100 pg/ml for PTX3 and 20 pg/ml for soluble IL-1RII. No cross-reaction with human CRP or serum amyloid P component was observed for antibodies used to detect PTX3.

Plasma level of IL-1 β was determined using commercially available kits (Quantikine HS High Sensitive ELISA [R&D Systems, Minneapolis, MN]). Sensitivity was 0.057 pg. /ml.

The concentration of all cytokines was determined by comparison with a standard curve, following the manufacturer's instructions.

### Statistical Analysis

The Shapiro–Wilk test was used to test the normal distribution of continuous variables. When continuous variables were normally distributed, the results were expressed as mean ± SD; otherwise, median and interquartile range (IQR; 25th- 75th percentile) were reported. Categorical variables were summarized as counts and percentages. Continuous variables were compared among groups (COPD patients, CHF patients, and healthy smokers) by ANOVA if normally distributed and by the Kruskal-Wallis test if non-normally distributed, with Bonferroni corrections for multiple testing. Categorical variables were compared among groups by the chi-square test or Fisher’s exact test, when appropriate. Correlation between continuous variables was assessed by using Spearman's rho. An ANOVA on ranks was constructed to compare IL-1β and sIL-1RII values among groups by considering potential confounders. P values <0.05 (two sided) were considered significant. Statistical analyses were performed using Stata version 12 (StataCorp LP, College Station, TX, USA).

## Results

### Clinical and Functional Characteristics of Study Groups

Seventy COPD patients, 124 CHF patients, and 24 healthy smokers (control subjects) were studied (Tables 1 and 2). CHF patients were slightly, but significantly older than both control subjects and patients with COPD. The percentages of males, BMI values, and number of pack years were similar in the three groups. Of the CHF patients, 86% were classified as New York Heart Association (NYHA) class I or II, and 63% of COPD patients were classified as GOLD stage I or II (Table 1). In the CHF group, 13 patients (11%) were treated with inhaled bronchodilators and 10 (8%) were treated with inhaled steroids (Table 1), as 34% of the CHF patients had airflow limitation. Of the CHF patients with airflow limitation, 52% were classified as GOLD stage I, 40% as GOLD II, and 8% as GOLD III. Patients with pure COPD had a higher 6MWT, a lower Charlson comorbidity index, a lower NT-proBNP, and a higher Hs-CRP compared with all the CHF patients (Table 2). None of the COPD patients showed impaired left ventricular systolic function (left ventricular ejection fraction [LVEF] ≤ 40%) or a left ventricular (LV) diastolic dysfunction. Likewise, we did not find levels of estimated systolic pulmonary artery pressure consistent with pulmonary hypertension. As mentioned above, 34% of CHF patients had airflow limitation. Partial arterial pressure of oxygen (PaO_2_) was higher and partial arterial pressure of carbon dioxide (PaCO2) was lower in CHF than in COPD (82.7 ± 10.9 vs. 75.1 ± 9.3 mm Hg, p < 0.001, and 38.8 ± 3.7 vs. 40.9 ± 4.5 mm Hg, p = 0.004, respectively). It is noteworthy that, while all the COPD patients underwent this measurement, 40% of the patients with CHF refused to perform it.

**Table 1:** Clinical characteristics of COPD patients, CHF patients, and healthy smokers (control subjects).

	**COPD**	**CHF**	**Healthy smokers**
	(n=70)	(n=124)	(n=24)
Age, yr*	68.7 ± 7.8	71.6 ± 6.9	67 ± 7.7
Males, n (%)	52 (74)	106 (86)	15 (62.5)
BMI, kg/m^2^	27.6 ± 4.6	28.1 ± 3.6	27 ± 5
Pack years	45.3 ± 27.1	41.8 ± 25.2	35.8 ± 15.4
GOLD stage, n (%)			
I	10 (14)	-	-
II	34 (49)	-	-
III	26 (37)	-	-
NYHA class, n (%)			
I	-	26 (21)	-
II	-	81 (65)	-
III	-	15 (12)	-
IV	-	2 (2)	-
Medication, n (%)			
ACE inhibitors	19 (27.5)	85 (68.5)	0
Beta blockers	14 (20)	103 (83)	0
Statins	20 (30)	79 (64)	0
Inhaled bronchodilators	57 (81)	13(11)	0
(LABA and/or LAMA)			
Inhaled steroids	43 (61)	10 (8)	0

Data are expressed as number of subjects (%) or mean ± SD.

Abbreviations: COPD, chronic obstructive pulmonary disease; CHF, chronic heart failure; BMI, body mass index; NYHA, New York Heart Association; GOLD, Global Initiative for Chronic Obstructive Lung Disease; ACE, angiotensin-converting enzyme; LABA, long-acting beta agonists; LAMA, long-acting muscarinic agonists;

* Significant (p < 0.05): COPD vs. CHF, and CHF vs. healthy smokers.

**Table 2:** Functional characteristics of COPD patients, CHF patients, and healthy smokers (control subjects).

	**COPD**	**CHF**	**Healthy smokers**	**p value**
	(n=70)	(n=124)	(n=24)	
Charlson comorbidity index	1 (1–2)	3 (2–4)	-	< 0.001
6MWT, m	490 ± 131	378 ± 163	N.A.	< 0.001
LVEF (%)	69.83 ± 7.04	40.45 ± 11.59	N.A.	< 0.001
NT-proBNP, pg/ml	115 (50–364)	984 (450–2095)	50 (43–51)	< 0.001*
Hs-CRP, mg/L	2.17 (0.93–4.62)	0.32 (0.20–0.70)	0.3 (0.17–0.55)	< 0.001**
Post-BD FEV1% predicted	60.48 ± 18.39	88.55 ± 20.26	115.77 ± 15.83	< 0.001***
Post-BD FVC % predicted	86.23 ± 20.85	94.04 ± 18.81	117.17 ± 16.11	< 0.001****
Post-BD FEV1/FVC ratio	0.54 (0.47–0.61)	0.74 (0.67–0.78)	0.77 (0.74–0.81)	< 0.001*****

Data are expressed as mean ± SD or median value (interquartile range: 25th–75th percentile).

Abbreviations: 6MWT, 6-min walk test; LVEF, left ventricular ejection fraction; NT-proBNP, N-terminal pro-hormone of brain natriuretric peptide; Hs-CRP, high-sensitive C-reactive protein; BD, bronchodilator; FEV1, forced expiratory volume in 1 s; FVC, forced vital capacity; N.A., not available.

* Significant (p < 0.05) post-hoc tests: COPD vs. CHF; COPD vs. healthy smokers; CHF vs. healthy smokers.

** Significant (p < 0.05) post-hoc tests: COPD vs. CHF; COPD vs. healthy smokers.

*** Significant (p < 0.05) post-hoc tests: COPD vs. CHF; COPD vs. healthy smokers; CHF vs. healthy smokers.

Significant (p < 0.05) post-hoc tests: COPD vs. CHF; COPD vs. healthy smokers; CHF vs. healthy smokers.

Significant (p < 0.05) post-hoc tests: COPD vs. CHF; COPD vs. healthy smokers; CHF vs. healthy smokers.

Hypertension (98%), myocardial infarction (58%), and hypercholesterolemia (35%) were the three most common comorbidities in CHF patients, whereas hypertension (50%), osteoporosis (14%), and diabetes (13%) were most common in COPD patients.

### PTX3, IL-1 β, and sIL-1RII

The plasma levels of PTX3 were similar in the three groups studied; in contrast, circulating IL-1 β was higher in COPD patients than in both CHF patients and control subjects (healthy smokers; p < 0.001). Plasma levels of IL-1 β did not differ between CHF patients and control subjects (Figure 1). Likewise, sIL-1RII systemic concentrations were significantly elevated in COPD compared to both CHF patients and control subjects (p < 0.05 and p < 0.01, respectively) (Figure 1).

**Figure 1:** PTX3 (A), IL-1β (B), and sIL-1RII (C) plasma levels in COPD, CHF and healthy smokers. IL-1β and sIL-1 RII plasma levels were significantly higher in COPD than in both CHF patients and control subjects (healthy smokers). PTX3 plasma levels did not differ among the three groups. Data are expressed as the median value; bars indicate the 75th and 25th percentiles. ○ p<0.001, COPD vs. CHF, and COPD vs. healthy smokers. *; p<0.05, COPD vs. CHF ; ** p<0.01, COPD vs. healthy smokers.

The potential correlations of PTX3, IL-1 β, and sIL-1RII with clinical variables (age, BMI, smoking pack years, GOLD stage, NYHA class, Charlson index, 6MWT, LVEF, NT-proBNP, Hs-CRP, FEV1 [% predicted], FEV1/FVC [forced vital capacity], and statin, inhaled bronchodilator and inhaled steroid treatments) were checked. PTX3 and sIL-1RII did not show clinically meaningful associations with any of those parameters. IL-1 β correlated negatively with NT-proBNP (rho = -0.34, p < 0.001), FEV1 (% predicted) (rho = -0.29, p < 0.01), and FEV1/FVC (rho = -0.35, p < 0.001), and correlated positively with Hs-CRP (rho = 0.30, p < 0.01).

Finally, an ANOVA on ranks was constructed to compare either IL-1 β or sIL-1RII values among groups, considering potential confounders such as age, smoking, pack years, NT-proBNP, Hs-CRP, FEV1 (% predicted), FEV1/FVC, and statin, inhaled bronchodilator and inhaled steroid medication. IL-1 β, but not sIL-1RII, remained significantly higher in COPD patients than in CHF patients and healthy smokers [1.43 (0.57-2.16) vs. 0.48 (0.34-0.88) and 0.47 (0.40-0.89, respectively, p < 0.0006].

## Discussion

Although we detected no echocardiographically documented CHF in well characterized smokers with COPD, we found airflow limitation in 34% of well-characterized smokers with CHF. Furthermore, we found evidence of low-grade systemic inflammation only in patients with COPD.

The finding of 34% airflow limitation in smokers with CHF is consistent with previously reported prevalences of COPD in patients with heart failure, ranging from 10 to 50% [17]. The prevalence of airflow limitation in our study was based on post-bronchodilator spirometry, whereas most of the previous studies were retrospective and COPD diagnosis was self-reported [10,11]. Notably, only 10 of our 42 patients with both CHF and COPD were aware of airflow limitation and were properly treated, highlighting the importance for better screening for this comorbidity in CHF patients [11].

Spirometry may be difficult to assess in elderly patients with CHF, and diagnosis of COPD may be under- or over-estimated in these patients. Spirometric abnormalities of the restrictive type may be present in patients with stable heart failure, and airflow limitation may develop in patients with decompensated heart failure [17]. Also, FEV1/FVC ratio might overestimate airflow limitation and thus over-diagnose COPD particularly in the elderly [18]. The “restrictive” abnormality might “mask” airflow limitation in stable CHF and thus cause under-estimation of airflow limitation and consequently underdiagnosis of COPD. By contrast, the transient airflow limitation might cause over-estimation of airflow limitation and consequently overdiagnosis of COPD in decompensated CHF. Even considering these limits of spirometry, it should be mentioned that spirometry is just one criterium for establishing the clinical diagnosis of COPD, the others being symptoms and risk factors (http://www.goldcopd.org/ .). Because the CHF subjects we examined were stable and were all smokers, we feel rather confident that the risk of misdiagnosis in this group of patients with CHF is limited.

We did not observe any overt LV systolic dysfunction (ie LVEF ≤40%) in COPD patients. Also LV end-diastolic size and LV end-systolic size were not abnormal in any but one patient with COPD, who had definitively increased LV end-diastolic and end-systolic diameters, according to the normal values indicated in the European Society of Cardiology guidelines for the diagnosis and treatment of acute and chronic heart failure [2]. The prevalence of left heart abnormalities previously described in COPD patients varies widely, from 0 to 32% [19,20], depending on whether the study was performed on selected patients with no history of coronary heart disease or on unselected subjects. In two recent studies, the prevalence of overt LV systolic dysfunction was 17% and 13%, respectively [20,21]. In the first survey [20], LV dysfunction burden was concentrated in COPD patients classified as GOLD III and IV (70%), with a significant proportion of subjects with documented ischemic heart disease (40.5%) and with a median value of NT-proBNP higher than that detected in our COPD population (677 vs. 115 pg/ml). Therefore, our failure to find left heart abnormalities might be explained by the different characteristics of our COPD patients. In the second study [21], the prevalence of overt LV systolic disfunction (LVEF < 40%) was < 4%, and the prevalence of impaired LV systolic function was present in 13% of subjects, although most often the impairment was mild (LVEF <0.50). 

The high LVEF (%) observed in our COPD might be explained by the following reasons: 1) patients with COPD were recruited in tertiary pulmonary referral centers, and were all on regular COPD pharmacologic treatment, and thus most likely patients with COPD and chronic heart failure were excluded from the recruitment; and 2) patients with COPD were all treated with long-acting bronchodilators associated or not with inhaled steroids, and thus the hemodynamic effects of the bronchodilator therapy may have contributed to the high values of LVEF. In fact both inhaled antimuscarinic and beta 2 agonist bronchodilators increase ejection fraction and stroke volume [22], 3) the result of a normal Nt-proBNP is consistent with the finding of a normal LVEF and excludes definitively a diagnosis of heart failure, either with reduced or preserved ejection fraction. In reality, heart failure is unlikely in patients showing a Nt-proBNP value less than 125 pg/ml, as reported in the diagnostic flowchart for suspected heart failure of the 2012 European Society of Cardiology guidelines [2]. 

It has been hypothesized that chronic low-grade systemic inflammation is a “common soil” for pulmonary and cardiovascular diseases, particularly COPD and CHF, and that aging, smoking, and obesity, the major risk factors for complex chronic disorders, cause systemic inflammation.

The results presented here show that the serum level of Hs-CRP was significantly higher in COPD patients than in CHF patients and control subjects, which did not differ from each other. The association between stable COPD and increased blood CRP is well established and helps to explain the presence of systemic inflammation in this chronic pulmonary disease [5]. In contrast, the role of inflammation in the pathogenesis of CHF is less well defined. There is evidence of elevated CRP levels in patients with heart failure in higher NYHA functional classes, with higher rates of hospital readmission and higher rates of mortality [6]. Our finding of a similar concentration of CRP in CHF patients and control subjects could be explained, at least in part, by the fact that most of the CHF patients in our study had stable, mild disease (NYHA classes I and II).

CRP is a member of the pentraxin superfamily. In recent years, another pentraxin, PTX3, has been investigated in both CHF and COPD. In CHF, PTX3 is related to more severe disease and worse outcomes, such as all-cause mortality, cardiovascular mortality, and hospitalization for decompensated heart failure [7]. Our study complements these previous observations by showing that the PTX3 plasma level of a cohort with mild symptomatic heart failure (NYHA classes I and II) and clinically stable heart failure is similar to that of healthy subjects matched for age and smoking history. With regard to COPD, we confirmed the earlier finding of circulating levels of PTX3 within the normal range [23]. 

IL-1 β, a proinflammatory cytokine, is increased in airway secretion during exacerbation of COPD [24,25] and correlates significantly with other inflammatory mediators and cells when COPD is stable [26]. Our finding of higher plasma concentrations of IL-1 β in COPD compared to control subjects (healthy smokers) is in agreement with the results of previous studies focused on profiling serum biomarkers in patients with stable COPD [27]. In contrast, this finding may appear to conflict with that of Sapey et al. [28], who found no differences in circulating IL-1 β between COPD patients and healthy subjects. However, they examined very few patients (n=15) and compared them with control subjects who had never smoked, making it impossible to distinguish between the effect of smoking and the effect of COPD.

Recent studies indicate that decoy receptors act as a general strategy to fine-tune the action of primary inflammatory mediators. The decoy receptor paradigm describes a receptor that is capable of recognizing its ligand with high affinity and specificity, but that is structurally incapable of signaling [29]. Soluble IL-1RII was the first pure decoy receptor to be identified, and, in the current study, we have shown that its systemic level is higher in COPD patients than in both control subjects and CHF patients. This increase may indicate an attempt to prevent the inflammatory biological effects mediated by the elevated IL-1 β in COPD patients. However, other investigations are better suited to clarify the role of sIL-1RII in COPD [28,30].

Circulating IL-1 β and sIL-1RII levels did not differ between our CHF patients and control subjects. This was not completely unexpected, as the inflammatory network in CHF is still debated. In particular, previous studies have reported that IL-1 β systemic levels in heart failure are either unchanged [31], increased [32], or decreased [33]compared to controls.

In conclusion, this report shows that airflow limitation is common and unrecognized in smokers with CHF, whereas a consistent impairment of LV function is not always detectable in well-characterized patients with COPD. In contrast to CHF patients, COPD patients show evidence of low-grade systemic inflammation, as demonstrated by an increase in CRP, IL-1 β, and sIL-1RII plasma levels. Better clinical and functional characterization of elderly smokers with chronic diseases, and identification of the key inflammatory mediators involved, may help to improve the treatment and management of these patients.
